The article "Management Cost Management and Resource Optimization of Construction Enterprises Based on Ecological Environment Constraints" was published in 2022. Journal: J Environ Public Health.

# Management Cost Management and Resource Optimization of Construction Enterprises Based on Ecological Environment Constraints

**DOI:** 10.1155/2022/9884746

**Published:** 2022-08-08

**Authors:** Yan Xing, Quanying Xin

**Affiliations:** College of Urban Construction, Hebei Normal University of Science and Technology, Qinhuangdao 066004, China

## Abstract

In recent years, with the proposal of the “One Belt, One Road” initiative, the domestic economy and its development have entered a new normal, which has promoted the determination and connection of the development strategies of various countries. It has brought new opportunities for the development of domestic enterprises. In this context, it has become a trend for Chinese enterprises to go international, especially in the construction industry; due to the good potential of the “Belt and Road” initiative, it is necessary to change and update from the traditional construction industry to modern construction industry. Therefore, how to promote the coordinated development of the construction company's resource management system, meet the needs of the company's own development, and adapt to the goals of internationalization and modern management have become a problem that people are very concerned about. The current domestic environmental situation is improving in part, but it is deteriorating in general. The harm caused by environmental pollution and damage is becoming more and more obvious. The construction industry is one of the national pillar industries, and it is also an industry with high energy consumption and high pollution. Based on this, this study first introduces construction enterprise management and resource optimization methods and integrates ecological environmental protection into enterprise operating cost management. Second, it establishes an enterprise-centric resource allocation model and optimization algorithm. An empirical study was carried out on the ecological management capabilities of three construction enterprises of different sizes, namely, Industrial Group, Group A, and Construction Enterprise B, and concluded that the overall level of environmental competitiveness of construction enterprises in my country is not high, among the environmental management and construction capabilities of enterprises. The standardization ability of ecological engineering construction is relatively weak, resulting in poor overall profitability of the enterprise, and the number of green suppliers does not meet the needs of ecological development. However, under the constraints of the ecological environment, construction enterprises compete with each other to control operating costs and at the same time affect the environment. At the same time, the allocation of resources by enterprises is also more conducive to the development of ecological civilization in the industry.

The article "Management Cost Management and Resource Optimization of Construction Enterprises Based on Ecological Environment Constraints" was published in 2022. Journal: J Environ Public Health.

## 1. Introduction

The dry land in western China refers to the vast area west of the Helan Mountains and north of the Kunlun Mountains. Studying and improving the ecological environment of the arid areas in this area are of great importance for the implementation of national strategies and policies to accelerate the development of the region and for maintaining social order and national territorial integrity [1]. The rise of nontectonic movement and climate warming and drying leads to the deterioration of ecological environment and the degradation of swamps. In addition, frequent human activities, including deforestation, draining swamps, exploiting peat, and overgrazing, make this possibility come true [2]. The combination of ecological vulnerability and agricultural activities in the loess hilly and gully region of western China has attracted extensive environmental concerns. The changes of soil moisture and fertilizer content at different depths in sloping farmland and terraced fields on the Loess Plateau were studied, and the ecological impact and economic benefits of terraced fields were evaluated [3]. Land consolidation is the reconstruction of the ecological environment system that affects regional environmental factors and ecological processes. There are three factors that affect the regional ecological environment in the process of land consolidation including the characteristics of land consolidation engineering, changes in land use types, and landscape pattern changes after land consolidation [4]. The level of marine environmental management is the key factor for the successful implementation of the strategy of marine power, and the improvement of the level of marine environmental management requires innovation in marine management. In other words, in order to realize the sustainable development of the marine economy, we must realize the transition from marine environmental management to marine ecological environment management [5]. In the construction industry, corporate social responsibility (CSR) is increasingly seen as a factor in promoting sustainable business operations. Based on stakeholder theory, CSR performance issues with different stakeholders are proposed to demonstrate the key factors of CSR performance in construction, and then indicators that reveal the content of performance issues are selected [6]. There are several possible paths of development for construction companies as they strive to grow. It has been found that most local contractors have grown up by working from home, either as a main contractor or as a specialist subcontractor, with advice on appropriate growth paths for Singaporean contractors in different contexts [7]. This paper proposes a method to determine the management strategy of construction enterprises. To this end, a SWOT (Strengths, Weaknesses, Opportunities, and Threats) analysis is recommended as a tool for developing a management strategy. Best practices in this regard are also analyzed. The algorithm is based on AHP, expert judgment, and feasible solution ranking method to select the optimal strategy [8]. In order to improve the performance of the construction industry, this paper analyzes the key factors that affect the effectiveness of organizational communication in construction enterprises and discusses the correlation between the effectiveness of organizational communication and alliance performance [9]. The construction industry is an important source of direct employment and, through its wide range of operations and projects, contributes to the growth and development of virtually every other sector of the economy. It is only from a pool of resourceful, well-trained, and motivated small contractors that well-founded mid-sized and larger local companies can gradually grow and grow [10]. The article explores how firms implement cross-organizational cost management in the product design process and the characteristics of the relational environment associated with it; it also discusses the impact of this development on making or purchase decisions [11], focusing on activity-based cost management (ABCM), which can provide better information for strategic decision-making in product planning and cost management, which is beneficial to the development and management of construction enterprises [12]. The cost of a relationship depends not only on the internal factors of both parties, but also on the level of focus with other relationships, so the way in which other parties (such as the supplier's other customers, the customer's other suppliers, and the customer's customers) affect the cost needs to be included in the under analysis [13]. We propose an autonomic computing approach to the problem of reconfiguration, enabling a service-based system to configure itself through a loop of monitoring, analyzing, planning, and executing actions [14]. Optima is a software package for epidemiological and intervention modeling that we developed to address practical policy and program problems encountered by funders, governments, health planners, and program implementers. Optima's key features are its the ability of performing resource optimization to meet strategic objectives, including associated financial commitment projections and health economic assessments [15].

The article "Management Cost Management and Resource Optimization of Construction Enterprises Based on Ecological Environment Constraints" was published in 2022. Journal: J Environ Public Health.

## 2. Construction Enterprise Management and Resource Optimization Methods

### 2.1. Status Quo of the Development of Domestic Construction Enterprises

In recent years, the situation of the domestic construction market has become more and more severe. From the global economic trend to the implementation of the government's new “National Five Regulations,” the current situation shows that the severe winter of the construction industry is coming again. The big environment is like this, the small environment is even less optimistic and it is difficult for ordinary local construction companies to maintain. Due to the low barriers to entry in the construction industry, nonlocal companies, small companies, partnerships, and even rural construction teams have begun to occupy certain markets, while local construction companies can only survive in the cracks; that is, they need to compete with large companies for financial resources and small units, price and the ability to compete with companies of the same size. In a word, in this case, it is not enough to only rely on financial resources, price, and interpersonal relationships to occupy the market and gain a certain market share; only well-run companies and project departments can have and manage absolute competitive advantages. In addition, project bids are more standardized, and checklist bids make project bids very transparent, making it more difficult to add costs and change the way in which costs go through standardized project management or design reviews. At the same time, in the context of such fierce competition, many construction companies continue to adopt a broad management model, and, in the long run, the company will fall apart. Therefore, enterprises and project departments must rely on advanced and efficient management models, low cost, and strict resource allocation in order to gain a firm foothold in the market and find a way to success.

### 2.2. Current Situation of Development of Foreign Construction Enterprises

A vast majority of construction companies in the United States, Japan, Britain, France, and other countries are statutory private companies with very few government shares and flexible labor systems. The workforce is mainly composed of contract agents or temporary workers, which are low-cost and flexible operating organizations. Internationally renowned construction companies can provide full-process management services in their engineering fields, limited not only to traditional construction contracts, but also to predesign, engineering, procurement, construction, commissioning, and operation services. According to the actual needs of the project, the company has the financial strength and advance payment ability. The company protects its long-term organizational interests through the industries that it serves, and, at the same time, it brings more added value to the organization by expanding its service areas.

The article "Management Cost Management and Resource Optimization of Construction Enterprises Based on Ecological Environment Constraints" was published in 2022. Journal: J Environ Public Health.

### 2.3. Ecological Environment Theory

According to Article 26 of the Constitution, the state protects and improves the ecological environment of residential areas and prevents environmental pollution and other hazards. In 2005, some academicians proposed the fact that the concept of “building an ecological environment” should be gradually revised. It can be said that the ecological environment is the environment, environmental issues such as pollution must be included, and they are inseparable. Some experts believe that the ecological environment should be defined as a more compatible ecological environment without major problems and other pollution, which can be understood as the sum of the material conditions for human survival and development.

#### 2.3.1. Human Resource Niche Theory

The precise content of the concept of human resource niche refers to the interaction and interdependence of organisms and their lives, as well as the environmental protection function of each other's systems. The interdependent human resources and environment objectively demonstrate the movement of all data flow transformations. Referring to and further refining the concept of HR niche in empirical research on companies, we first discuss HR management systems and further define the concept of HR niche: the precise location of an individual (or group) in a specific environment. In addition to the fact that it mainly expresses personal development and viability, it also contains other environmental factors.

#### 2.3.2. The Path to Optimize the Human Resources Ecological Environment of Construction Enterprises

Use the design hypothesis model to extensively analyze human resources, evaluate the internal relationship of environmental and environmental factors, build the company's human resources ecological evaluation system, conduct a comprehensive evaluation of the ecological environment of the construction enterprise, combine the evaluation specific practice, and set optimization measures to achieve the expected research goals.

### 2.4. Enterprise Resource Optimization Methods

There are many research methods on the balanced allocation of corporate resources at home and abroad:

1. Manual method: this method is intuitively realized from the network diagram of the project on the basis of the CPM method, also known as the graphical method, but this method has obvious shortcomings and is only suitable for simple network diagrams. The scale of the project increases, the amount of calculation and the difficulty increases greatly, and the optimization cannot be achieved by artificial methods. Although this method produces a balanced solution with a smaller grid size, it is difficult to achieve the optimal guarantee.
2. Mathematical programming method: in theory, no matter how complex the network graph is, the resource balance problem can always be determined by mathematical methods and then solved by existing linear programming methods. However, when there are too many programs in a project, and the relationships between them are complex, there are too many variables and constraint equations related to the problem, and the feasibility becomes poor.
3. Heuristic method: with the deepening of the research and application of intelligent algorithms, many researchers use this idea to solve the problem of resource balance, such as tabu search algorithm and simulated luminescence algorithm. These methods are algorithms for finding the solution space according to certain rules. This method has a fast convergence speed and can quickly obtain the optimal solution.

The article "Management Cost Management and Resource Optimization of Construction Enterprises Based on Ecological Environment Constraints" was published in 2022. Journal: J Environ Public Health.

## 3. Enterprise Center Resource Allocation Model and Optimization Algorithm

### 3.1. Convex Optimization Theory

In convex optimization research, the minimization problem of convex function defined by convex set is an important part of mathematical optimization research, and the most common problem form is mainly linear programming problem. In general, convex optimization problems have the following form:

(1) $$\begin{array}{c} \min f_{0}\left(x\right),\\ \text{subject to }f_{i}\left(x\right)\leq b_{i},\;i=1,\ldots ,m\\ a_{i}^{T}=b_{i},\;i=1,\ldots ,p. \end{array}$$

Among them, the function is a convex function, the convex optimization problem must satisfy the inequality constraint function that must be a convex function, and the equality constraint function *h*_*i*_(*x*)=*a*_*i*_^*T*^ − *b*_*i*_ must be an affine function.

### 3.2. Lagrangian Dual Function

Consider an optimization problem of the following standard form:

(2) $$\begin{array}{c} \min f_{0}\left(x\right),\\ \text{subject to }f_{i}\left(x\right)\leq 0,\;i=1,\ldots ,m\\ {\text{h}}_{i}\left(x\right)=0,\;i=1,\ldots ,p. \end{array}$$

The basic idea of Lagrangian duality is to emphasize the limitation of formula (2) and add it to the objective function to obtain the optimal function. The above optimization problem can be expressed in the following form:

(3) $$\begin{array}{c} L\left(x,\lambda ,v\right)=f_{0}\left(x\right)+\sum_{i=1}^{m}\lambda_{i}f_{i}\left(x\right)+\sum_{i=1}^{p}v_{i}h_{i}\left(x\right), \end{array}$$

where the vectors *λ* and *v* are called binary variables or Lagrange multiplier vectors of formula (2). Define Lagrangian dual function:

(4) $$\begin{array}{c} g\left(\lambda ,v\right)=\underset{x\in s}{\min}L\left(x,\lambda ,v\right). \end{array}$$

If a Lagrangian function has no lower bound on x, its double-precision function has the value −*∞*. For any set (*λ*, *v*), the Lagrangian bifunction forms a lower bound on the maxima of the optimization problem as follows:

(5) $$\begin{array}{c} g\left(\lambda ,v\right)\leq p^{*}. \end{array}$$

The Lagrangian double function can be expressed as the following optimization problem:

(6) $$\begin{array}{c} \max g\left(\lambda ,v\right),\\ \text{subject to }\lambda \geq 0. \end{array}$$

The set (*λ*, *v*) that satisfies the conditions is called a feasible solution, and the solution obtained after the objective function of equation (6) reaches the maximum value is the optimal solution of the dual problem, which can be expressed as (*λ*^*∗*^, *v*^*∗*^).

The article "Management Cost Management and Resource Optimization of Construction Enterprises Based on Ecological Environment Constraints" was published in 2022. Journal: J Environ Public Health.

Regardless of whether the original problem is a convex optimization problem, the double Lagrangian function is a convex optimization problem. In an optimization problem, when the constraints are difficult to solve for the optimal value of the optimization problem, it can be solved neatly.

### 3.3. Construction of the Central Resource Allocation Model

The purpose of allocating resources is to use the resources of an appropriate amount of physical machines as efficiently as possible. For this reason, the following optimal resource allocation models for cloud virtual server centers are constructed:

(7) $$\begin{array}{c} \max\sum_{s\in s}U_{s}\left(y_{s}\right) \end{array}$$

(8) $$\begin{array}{c} \text{over }x_{sr}^{\min}\leq x_{sr}^{p}\leq x_{sr}^{\max},r\in R,s\in S,p\in P. \end{array}$$

For the fairness of virtual machine resource allocation in the enterprise private cloud, selecting the appropriate tool may result in the corresponding resource allocation. Consider the following useful functions:

(9) $$\begin{array}{c} U_{s}\left(y_{s}\right)=W_{s}\log\;y_{s}. \end{array}$$

Among them, *W*_*s*_ is the voluntary payment of cloud users in the enterprise in order to obtain the corresponding resource allocation when configuring parameters.

#### 3.3.1. Model Analysis

For the resource allocation model (7) and its utility function (9) proposed in this paper, the objective function is strict for *y*_*s*_; although *x*_*sr*_^*p*^ is not a strictly convex function, under linear constraints, the convex set is an allocation of resource-constrained optimal sets. The following results can be obtained from the convex optimization theory. In order to obtain the optimal solution of the enterprise resource allocation model, the Lagrangian function is introduced.

(10) $$\begin{array}{c} L\left(x,y,\lambda ,\mu \right)=\sum_{s\in S}\left(U_{s}\left(y_{s}\right)-\lambda_{s}y_{s}\right)+\sum_{pr}\sum_{s}x_{sr}^{p}\left(\left(\lambda -\mu_{p}\right)+C_{p}\right). \end{array}$$

Among them, *λ*=(*λ*_*s*_, *s* ∈ *S*) is the payment that enterprise cloud users pay for each unit of computing resources. Price*μ*=(*μ*_*p*_, *p* ∈ *P*) is the fee charged per unit of PM computing resources in

(11) $$\begin{array}{c} S_{s}\left(\lambda_{s}\right)=\max U_{s}\left(y\right)-\lambda_{s}y_{s}, \end{array}$$

(12) $$\begin{array}{c} P_{ps}\left(\lambda_{s},\mu_{p}\right)=\max x_{sr}^{p}\left(\lambda -\mu \right). \end{array}$$

In (11), enterprise cloud users attempt to maximize value based on the total resources obtained depending on their role in deploying the application cloud. In (12), the application component extracts the resource configuration value *x*_*sr*_^*p*^ from the physical machine. Since physical machines offer a price per resource unit, the cost value of resource value is allocated to physical machines, so (12) shows that PM maximizes its own benefit; the following is a duplicate of how to solve the virtual machine resource allocation problem:

(13) $$\begin{array}{c} \min\;D\left(\lambda ,\mu \right),\\ \text{subject to }\lambda_{s}\geq 0,\mu_{p}\geq 0. \end{array}$$

Problem (7) is to maximize the overall efficiency of cloud applications under the limited PM resources of the enterprise cloud service center, while problem (13) is to minimize the total cost of cloud services. When deploying applications in the cloud, in order to obtain the optimal allocation of virtual machine resources, whether it is the optimal solution of the original problem or the repeated problem, we get

(14) $$\begin{array}{c} y_{s}^{*}=\frac{W_{s}}{\lambda_{s}}. \end{array}$$

It can be seen that the total resource configuration value obtained by the VM where each application is located is unchanged. In addition, according to the different resource configuration requirements of enterprise cloud service users, other types of auxiliary functions can be selected to realize different types of auxiliary functions to resource allocation goals.

The article "Management Cost Management and Resource Optimization of Construction Enterprises Based on Ecological Environment Constraints" was published in 2022. Journal: J Environ Public Health.

### 3.4. Central Resource Allocation Algorithm

To understand whether the virtual machine where each application's components are located can perform resource optimal allocation when enterprise cloud users deploy applications in the cloud, this paper proposes the following enterprise resource allocation algorithm:

(15) $$\begin{array}{c} \frac{d}{dt}x_{sr}^{p}\left(t\right)=\theta x_{sr}^{p}t\left(\lambda_{s}\right)-\varepsilon \left(t\right), \end{array}$$

(16) $$\begin{array}{c} \varepsilon \left(t\right)=\frac{\sum_{j\in s\left(p\right)}\sum_{i\in R\left(j\right)}x_{ji}^{p}\left(t\right)\lambda_{j}\left(t\right)}{C_{p}}. \end{array}$$

The process-specific prices that corporate cloud users pay for deploying cloud applications are

(17) $$\begin{array}{c} \lambda_{s}\left(t\right)=\frac{W_{s}}{\max\left\{\eta ,y_{s}\left(t\right)\right\}}, \end{array}$$

(18) $$\begin{array}{c} y_{s}\left(t\right)=\min\left\{y_{s}^{\max},\max\left(\sum_{rp}x_{sr}^{p}\left(t\right),y_{s}^{\min}\right)\right\}. \end{array}$$

In the above algorithm, the expected price of the physical machine can be regarded as the supply of resources, and the expected price of the physical machine at the equilibrium point is equal to the price actually paid by the user.

#### 3.4.1. Resource Allocation Algorithm

When considering this function tool, the following enterprise resource allocation algorithm is recommended to achieve optimal resource allocation for each enterprise encapsulating the application when the enterprise cloud user deploys the application in the cloud:

(19) $$\begin{array}{c} \frac{d}{dt}x_{sr}^{p}\left(t\right)=\theta x\left(t\right)\left(\lambda_{s}t-\varepsilon_{pt}\right), \end{array}$$

(20) $$\begin{array}{c} \varepsilon_{p}\left(t\right)=\frac{\sum_{ji}x_{ji}^{p}\left(t\right)\lambda_{j}\left(t\right)}{C_{p}}, \end{array}$$

(21) $$\begin{array}{c} \lambda_{s}\left(t\right)=\frac{W_{s}}{\max\left\{\eta ,y^{\alpha }\left(t\right)\right\}}. \end{array}$$

In the above algorithm, *ε*_*p*_(*t*) can be considered as the expected price payment when the physical machine provides resources. At the equilibrium point, the expected price of the physical machine is the same as the price actually paid by the user.

### 3.5. Algorithm Implementation

In a particular implementation of an algorithm, resource allocation is made according to the discrete expression of the algorithm. That is, at time t = 1, 2, each corporate sector p allocates resources according to the following expression.

(22) $$\begin{array}{c} x_{sr}^{p}\left[t+1\right]=\left(\left(1-\varsigma \right)x_{sr}^{p}\left[t\right]+\varsigma \theta x^{p}\left[t\right]\left(\lambda_{s}\left[t\right]-\varepsilon_{p}\left[t\right]\right)\right), \end{array}$$

(23) $$\begin{array}{c} \bar{x_{sr}^{p}}\left[t+1\right]=\left(1-\varsigma \right)x_{sr}^{p}\left[t\right]+\varsigma x_{sr}^{p}\left[t\right]. \end{array}$$

Additional variables are introduced here, which are considered to be estimates of the optimal allocation of resources. Low-pass filtering is a filtering method. Through low-pass filtering, the algorithm fluctuation phenomenon is caused by the fact that the model is not strictly convex optimization and the optimal allocation of resources is not necessarily unique. Therefore, a low-pass filter model can be added to the original algorithm. The price paid for each application depends on the algorithms given in (17) and (18). In this chapter, a resource allocation model is designed to maximize server availability in a cloud environment, and the model is analyzed. After the analysis, specific expressions are obtained to optimize the resource allocation for each application. According to the resource allocation model, the optimal allocation of resources in the enterprise cloud service center is realized, and the convergence and stability of the algorithm are explained by using the optimization theory and stability theory.

The article "Management Cost Management and Resource Optimization of Construction Enterprises Based on Ecological Environment Constraints" was published in 2022. Journal: J Environ Public Health.

## 4. Empirical Research on the Management of Construction Enterprises in the Ecological Environment

### 4.1. Enterprise Selection

#### 4.1.1. Shanghai Construction Engineering Group

Shanghai Construction Engineering Group is an industry-leading construction enterprise with total assets of 195.7 billion yuan. It consists of five departments: construction, construction, real estate development, design consulting, and urban construction. The company's business covers dozens of countries and regions in Asia, Africa, and Europe, ranking 9th in the “World's Largest 250 International Design Contractors” in 2018. R&D investment was 4.6 billion yuan, accounting for 3.24% of operating income, and there were 6,719 R&D activities. The total number of scientific researchers is 6,719, accounting for 19.2% of the total number of employees, and about 80% are university graduates. It has 1 national-level enterprise technology center and several technology research centers to develop new products for the company. It also has many high-tech companies. According to the 2017 financial statements released by Shanghai Construction Engineering Group, the company's operating profit in 2017 was about 142.1 billion yuan, a considerable increase from the total profit of the previous year. In recent years, the company's business has continued to grow, which is reflected in the fact that the value of newly signed contracts in 2017 increased by one-fifth over the previous year, of which the construction industry accounted for more than half of the annual contract value.

#### 4.1.2. Group A

Group A is an unlisted group company. Relevant information is collected from the inside. The group has various general contracting qualifications for smelting, housing, municipal, steel structure, electromechanical, and road infrastructure projects. The company has total assets of 1.58 billion yuan and thousands of employees. A third of them have a university degree or higher, and they mainly work on domestic construction projects. In recent years, the average operating income of the enterprise is nearly 10 billion yuan, and the total profit is 200 million yuan. The annual investment in technology research and development and technology introduction accounts for more than 20% of the profit.

The article "Management Cost Management and Resource Optimization of Construction Enterprises Based on Ecological Environment Constraints" was published in 2022. Journal: J Environ Public Health.

#### 4.1.3. Construction Company B

Construction Company B is a company engaged in general contracting activities of construction projects. It has the second-level general contracting qualifications for housing construction projects and the second-level general contracting for mechanical and electrical installation projects. The total assets are 40 million yuan. In 2017, the company's operating profit was about 50 million yuan, and the total profit only accounted for 1 million yuan. The company has a total of 400 employees, including 97 juniors. The total number of action items in 2018 was 8, of which the national environmental inspector found that the company had caused great damage to the surrounding environment and there was no specific rectification in between. As a result, many migrant workers left the project, resulting in a shortage of project and late construction personnel. In the field of technology research and development and implementation, only about 200,000 yuan per year was sent to relevant operators to study and train abroad and won the Bashu Cup and Tianfu Cup.

### 4.2. Analysis of Ecological Competitiveness

This time, three types of construction companies of different sizes were selected for case studies. One is a large enterprise with a large business park and is listed on the stock exchange. This article chooses Shanghai Construction Engineering Group as the representative of such a company; the other is a company in the middle of the industry. Here, Group A is a good representative of the A type of company, a type of small business that basically survives the gap. In this article, B Construction Company was chosen to represent these types of companies.

According to the evaluation criteria of each single factor, 3 companies were investigated, respectively, and 15 domain experts who knew about these 3 companies were interviewed by means of a questionnaire survey. The results of the study are listed in Tables 1–3.

X11 indicates the ability of dealing with policies and laws, X12 indicates the ability of dealing with market risks, X61 indicates the degree of cultural integration of the project, and X62 indicates the greenness of green building products. The evaluation results of Tables 1 and 3 show that Shanghai Construction Engineering Group is much stronger than the other two companies in terms of its ability of dealing with policies and laws and market risks. Construction companies are average in all aspects, especially in terms of greenness of green building products and implementation of environmental protection measures. The reason may be that smaller companies are relatively lacking management costs and ecological protection awareness.

The article "Management Cost Management and Resource Optimization of Construction Enterprises Based on Ecological Environment Constraints" was published in 2022. Journal: J Environ Public Health.

### 4.3. Weight Analysis of Indicators at All Levels

This article is honored to invite 10 experts with rich experience in the construction industry to participate in the index analysis of this survey, including 7 masters and more than 4 with more than 10 years of industry experience. Each indicator score is designed to be 100 points. First, reliability tests are performed on different index layers and different module layers of the returned query data. The test results are shown in Figure 1. The reliability tests are all greater than 0.7, indicating that the data information is good and suitable for this study.

The Cronbach's alpha coefficient is a statistic and is the most commonly used measure of reliability. If the alpha coefficient reaches 0.7–0.8, it means that the scale has considerable reliability, and when it reaches 0.8–0.9, it means that the reliability of the scale is very good. X represents the competitiveness of enterprise ecological management, X1 represents the ability of the enterprise of dealing with the external environment, X2 represents the ecological capital capability, X3 represents the ecological management and construction capability, X4 represents the ecological construction standardization capability, X5 represents the implementation of ecological construction measures, and X6 represents the ecological product capability. The test results show that the environmental competitiveness of Shanghai Construction Engineering Group is at an excellent level, the environmental competitiveness of Group A is at a medium level, the environmental competitiveness of Construction Company B is at a poor level, and the environmental competitiveness of most companies is at a disadvantage. The weight of each indicator is calculated according to Table 4.

It can be seen from Table 4 that the competitiveness of enterprises in ecological management is slightly higher than the competitiveness of ecological project construction and the ability of ecological capital is slightly more important than the ability of dealing with the external environment and the ability of managing and constructing ecological financial risks. In the competitiveness of project ecological construction management, the ability of regulating ecological construction is more important than the ability of implementing ecological construction measures and the ability of ecological products. Ecological building standardization can solve all the problems that may arise in the construction process. It is an effective environmental protection method for enterprises to improve construction efficiency and monitor construction safety and progress.

The article "Management Cost Management and Resource Optimization of Construction Enterprises Based on Ecological Environment Constraints" was published in 2022. Journal: J Environ Public Health.

According to the set single-factor evaluation, the comprehensive evaluation results are divided into four grades: excellent, good, medium, and poor, and the corresponding score ranges are 100-90 points, 90-80 points, 80-70 points, and 70-60 points. The comprehensive assessment results of Shanghai Construction Engineering Group, Group A, and Company B were scored, with 95 points, 85 points, 75 points, and 65 points as the medians, respectively. The calculation results are shown in Figure 2. The comprehensive environmental competitiveness of Shanghai Construction Engineering is 87 points, that of Group A is 77 points, and that of Company B is 63 points.

From the comparison of the comprehensive evaluation results of the three groups in Figure 2, it can be concluded that Shanghai Construction Engineering Group invested a lot of money to protect and control the pollution of production waste, while Construction Group B did not meet the standards in the environmental inspection.

### 4.4. Analysis of Evaluation Results

The environmental competitiveness evaluation of Shanghai Construction Group is excellent. Among them, the company has strong environmental management capabilities, good project ecological construction, and the company's environmental competitiveness is the strongest. Shanghai Construction Engineering Group attaches great importance to ecological talents and capacity building. Ecological technology research and development and innovation enterprises should increase ecological assessment and monitoring. The ecological construction competitiveness of the project is weak, among which the standardization of ecological construction is average, the implementation of ecological measures is good, and ecological products have certain competitive advantages (see Figure 3).

*A*. The environmental competitiveness of the enterprise is at the average level, the enterprise environmental management competitiveness is very poor, the project ecological construction competitiveness is slightly stronger than the company's environmental management, the external response ability is relatively strong, and the company's environmental management and construction are average and the proportion of ecological personnel and green suppliers. The ratio is low, the company's environmental capital capacity is poor, and the balance sheet total and profit margin are not high. In the ecological construction competition of the project, the structural standardization ability is at a good level, and the ecological measure implementation ability standardization ability is the weakest (Figure 4).

The article "Management Cost Management and Resource Optimization of Construction Enterprises Based on Ecological Environment Constraints" was published in 2022. Journal: J Environ Public Health.

*B.* The environmental competitiveness of construction enterprises is poor, the ability of enterprises of dealing with the external environment and ecological capital in the competitiveness of enterprise environmental management is at a general level, and the ability of enterprise environmental management and construction is also poor. The ratio between ecotalents and ecotech investments is seriously insufficient. The environmental protection in the construction process is not considered, there is a clear lack of green suppliers, and the project's environmental management capabilities are poor (as shown in Figure 5).

Judging from the weighted total score, Shanghai Construction Engineering Group has the strongest environmental competitiveness, followed by Group A, and Construction Engineering Enterprise B is the weakest. Most of the companies are still in the position of A Company and Construction Company B, which shows that the overall environmental competitiveness of my country's construction companies is not high. The results of case analysis show that the ecological development of my country's construction enterprises has problems such as ecological capital, weak operation and construction capabilities, and weak ecological construction standardization capabilities.

### 4.5. Research Conclusions

1. In terms of environmental management, due to the company's low profit margin, low ability of protecting the environment, and low investment in green technology, the company's ecological capital and management and construction capabilities are relatively weak. The profit rate of Shanghai construction enterprises is 2.27%, the profit rate of Company A is 1.95%, and the profit rate of Construction Company B is 2.5%, which is significantly lower than that of other industries. The number of green suppliers obviously does not meet the company's environmental protection development needs. The ratio of environmental capabilities to ecological technology investment in two companies A and B is obviously insufficient, resulting in insufficient ecological environment management and construction capabilities of the company.
2. The main problem in the ecological construction of the project is that the standardization ability of ecological construction is weak and it is difficult to improve the efficiency of ecological construction. The ecological construction competitiveness of Shanghai Construction Engineering Group's projects is weaker than the standardization level of ecological management construction, but the implementation of ecological measures is good, and ecological products have certain competitive advantages. The standardization of construction of enterprise A is proportional to the implementation of ecological measures and the ability of ecological products is relatively weak, and the ecological competition position of Construction Company B is generally poor.

The article "Management Cost Management and Resource Optimization of Construction Enterprises Based on Ecological Environment Constraints" was published in 2022. Journal: J Environ Public Health.

## 5. Conclusion

This paper examines the ecological management of enterprises from the perspective of ecological environmental protection and green economy. The ecological management of enterprises is the starting point of the competitiveness of enterprises' normal production and operation. Through the research on the characteristics of construction enterprise management and its related sustainable competitiveness and green competitiveness, the connotation of construction enterprise ecological management is getting stronger and stronger. The competition of ecological engineering construction is the competition of ecological efficiency. The empirical research on the ecological management of construction enterprises shows that the ecological competitiveness of construction enterprises in my country is not high and the enterprises usually have problems such as low profitability and the number of green suppliers that do not meet the needs of ecological development. In response to these problems, we recommend that construction companies protect the ecological environment, achieve mutual benefit and win-win, long-term sustainable development, build an ecological supply chain, and improve the quantity and quality of buildings. At the same time, they formulate standards to improve the technological innovation ability of enterprises and improve the standardization ability of ecological construction. In practice, it is conducive to improving the ecological management capabilities of enterprises, conducive to ecological transformation of construction enterprises, and conducive to the construction of ecological civilization in the industry. The number of samples in this study can be further enriched, and the number of samples can be increased in subsequent studies. The enterprise resource model constructed this time conducts research on the operating cost of construction enterprises, and the results are subject to certain subjectivity. In the follow-up research, the model can be optimized to improve the objectivity of the evaluation results.

## Figures and Tables

**Figure 1:** Cronbach a reliability test of each index layer.

The article "Management Cost Management and Resource Optimization of Construction Enterprises Based on Ecological Environment Constraints" was published in 2022. Journal: J Environ Public Health.

**Figure 2:** Comparison of the comprehensive evaluation results of the three groups.

**Figure 3:** Comparison results of secondary indicators of Shanghai Construction Engineering Group.

**Figure 4:** Comparison results of the secondary indicators of Group A.

**Figure 5:** Comparison results of secondary indicators of construction enterprises in B.

**Table 1:** Evaluation results of the ecological competitiveness of Shanghai Construction Engineering Group.

Evaluating indicator	Outstanding	Good	Same as
X11	1	0	0
X12	0.9	0.1	0
X31	0.3	0.6	0.1
X32	0.4	0.4	0.2
X41	0.25	0.25	0.5
X42	0.35	0.2	0.45
X51	0.35	0.65	0
X52	0.15	0.1	0.75
X61	0.4	0.25	0.35
X62	0.35	0.35	0.3

**Table 2:** A group's ecological competitiveness evaluation results.

Evaluating indicator	Outstanding	Good	Same as	Range
X11	0.55	0.15	0.3	0
X12	0.55	0.45	0	0
X31	0.1	0.35	0.55	0
X32	0	0.1	0.65	0.25
X41	0	0.1	0.15	0.75
X42	0.4	0.6	0	0
X51	0	0	0.85	0.15
X52	0.15	0	0.85	0
X61	0.1	0.7	0.2	0
X62	0	0	0.65	0.35

**Table 3:** B group' evaluation results of ecological competitiveness of construction enterprises.

Evaluating indicator	Outstanding	Good	Same as	Range
X11	0	0	0.35	0.65
X12	0	0.3	0.55	0.15
X31	0	0	0.3	0.7
X32	0	0	0.35	0.65
X41	0	0.1	0.7	0.2
X42	0	0	0.35	0.65
X51	0	0	0.3	0.7
X52	0	0.25	0.55	0.2
X61	0	0.55	0.25	0.2
X62	0	0.1	0.15	0.75

**Table 4:** Weights of evaluation indicators for ecological competitiveness of construction enterprises.

Evaluating indicator	Secondary index weight	Level 3 index weight
X11	0.3021	0.4976
X12	0.5254	0.5024
X31	0.3656	0.2092
X32	0.3323	0.1992
X41	0.3860	0.4965
X42	0.3216	0.5035
X51	0.2924	0.2125
X52	0.4746	0.2013
X61	0.5567	0.5050
X62	0.2379	0.4950

## Data Availability

The data used to support the findings of this study are available from the corresponding author upon request.
